The article "Exploring the Muscle Metabolomics in the Mouse Model of Sepsis-Induced Acquired Weakness" was published in 2022. Journal: Evid Based Complement Alternat Med.

# Exploring the Muscle Metabolomics in the Mouse Model of Sepsis-Induced Acquired Weakness

**DOI:** 10.1155/2022/6908488

**Published:** 2022-08-16

**Authors:** Yikang Jiang, Qiang Wei, Wei Liu, Qiunan Chen, Xia Chen, Zhongzhen Yuan, Na Luo, Xi Chen, Chuanjiang Wang

**Affiliations:** ^1^Department of the First Clinical College, Chongqing Medical University, Chongqing, China; ^2^Department of Laboratory Medicine, The First Affiliated Hospital of Chongqing Medical University, Chongqing, China; ^3^Department of Orthopaedic Surgery, The First Affiliated Hospital of Chongqing Medical University, Chongqing, China; ^4^Department of Critical Care Medicine, The First Affiliated Hospital of Chongqing Medical University, Chongqing, China; ^5^Department of Health Management, Army Medical Center of PLA, Chongqing, China; ^6^Department of Pharmacy, Chongqing University Cancer Hospital, Chongqing Cancer Institute, Chongqing Cancer Hospital, Chongqing, China

## Abstract

**Background/Aim:**

We aimed to identify the differentially expressing metabolites (DEMs) in the muscles of the mouse model of sepsis-induced acquired weakness (sepsis-AW) using liquid chromatography-mass spectrometry (LC-MS).

**Materials and Methods:**

Sepsis by cecal ligation puncture (CLP) with lower limb immobilization was used to produce a sepsis-AW model. After this, the grip strength of the C57BL/6 male mice was investigated. The transmission electron microscopy was utilized to determine the pathological model. LC-MS was used to detect the metabolic profiles within the mouse muscles. Additionally, a statistically diversified analysis was carried out.

**Results:**

Compared to the sepsis group, 30 DEMs, including 17 upregulated and 13 down-regulated metabolites, were found in the sepsis-AW group. The enriched metabolic pathways including purine metabolism, valine/leucine/isoleucine biosynthesis, cGMP-PKG pathway, mTOR pathway, FoxO pathway, and PI3K-Akt pathway were found to differ between the two groups. The targeted metabolomics analysis explored significant differences between four amino acid metabolites (leucine, cysteine, tyrosine, and serine) and two energy metabolites (AMP and cAMP) in the muscles of the sepsis-AW experimental model group, which was comparable to the sepsis group.

**Conclusion:**

The present work identified DEMs and metabolism-related pathways within the muscles of the sepsis-AW mice, which offered valuable experimental data for diagnosis and identification of the pathogenic mechanism underlying sepsis-AW.

## 1. Introduction

Sepsis is referred to as a systemic inflammatory response syndrome and results from organ injuries caused by infections [1]. It is one of the leading causes of in-hospital mortality in the intensive care unit (ICU), with the mortality rate being 30–50% [2]. Besides the functional damage caused to important organs (such as kidneys and lungs) by macrocirculation or microcirculation, the dysfunctions of skeletal muscle, lymphocytes, etc., traditionally referred to as nonvital organs, can also occur at the same time [3]. Among these, the dysfunction of skeletal muscle develops rapidly, causing ICU-acquired weakness (ICU-AW), which in turn, affects the prognosis of sepsis patients [4, 5]. Studies have shown that acquired myasthenia is a common complication among sepsis cases, and its severity is tightly associated with the severity of sepsis [6]. During sepsis, massive inflammatory mediators and toxins are released, which cause ischemia/hypoxia injury due to the disturbance in microcirculation [7]. This activates the protease system and oxidative stress, which leads to dysfunction in mitochondria and changes in ion channels [8]. The entire process jointly constitutes the basis of neuromuscular diseases, which results in a decreased excitability of central nerves, peripheral nerves, and sarcolemma along with the changes in the neuromuscular junction [9]. This causes skeletal muscle contraction disorder, promoting the occurrence and development of acquired myasthenia [9]. Although sepsis-related deaths have shown a decreasing trend in the past decades, with some patients surviving the critical disease, most of them result in seriously limited functions [10]. Typically, a major limitation encountered by ICU survivors is the continued weakness of the skeletal muscle [11]. Even after the sepsis resolves, the symptoms of skeletal muscle weakness may last for many years in several cases (e.g., continued impairments related to neuropsychological disorders, posttraumatic stress disorder, bilateral forefoot dysfunction due to vasopressor use, etc.) [12]. The weakness of the skeletal muscle can also result in death [13]. Currently, there are limitations in the clinical assessment of sepsis-acquired muscle weakness. The medical research council score (MRC-score) has been used widely to assess and diagnose acquired myasthenia [14]. However, this method has major limitations and it also requires the patient to be sufficiently awake to cooperate with the examination [15]. Therefore, diagnosing and managing sepsis-associated acquired myasthenia is a challenge for ICU clinicians due to a lack of specific detection methods.

The article "Exploring the Muscle Metabolomics in the Mouse Model of Sepsis-Induced Acquired Weakness" was published in 2022. Journal: Evid Based Complement Alternat Med.

Metabolomics involves the entire chemical responses occurring inside the cells. It has been considered a strong global platform used to identify and quantify low-molecular-weight (LMW) metabolites within the biological samples [16]. Metabolism involves direct responses to the microenvironment, while the markers for metabolites may provide several other inputs (environmental, transcriptional, and translational) [17]. Recently, metabolomics has been used widely for the contemporary medical treatment of sepsis [18]. During the study of sepsis-related encephalopathy, metabolomics was used to analyze the characteristic metabolic biomarkers (4 -hydroxyphenylacetic acid) and specific metabolic pathways (ornithine cycle, etc.). These could indicate an early warning sign for septic encephalopathy [19]. Lin et al. found gas chromatography-mass spectrometry (GC-MS) to be the possible metabolomics approach for exploring sepsis and associated organ dysfunction [20]. During septic kidney injury, metabolites such as asymmetric dimethylarginine (ADMA) and adenosine triphosphate (ATP) could be used as specific biomarkers [21]. Therefore, metabolomics may reflect the internal environment and indicate particular usefulness in the identification of septic biomarkers for organ injury.

This study adopted the sepsis-acquired myasthenia experimental animal model established by Bassem Habr [22] et al. At first, we evaluated the potential metabolic phenotype of sepsis-acquired myasthenia by investigating different metabolic statuses between the skeletal muscles in normal control, sepsis, and sepsis-acquired myasthenia groups. Second, targeted and untargeted metabolomics approaches were used to identify the alterations in metabolites and metabolism-related pathways associated with sepsis-mediated muscle weakness. Thus, we aimed to shed light on novel markers of early diagnosis and treatment of sepsis-mediated myasthenia.

## 2. Materials and Methods

### 2.1. Ethical Approval

This study was approved by the Ethics Committee of the First Affiliated Hospital of Chongqing Medical University (Approval number: 2020–845). All animals were treated as per the guidelines of Laboratory Animal Care and Use in China. The study protocols were approved by the Institutional Animal Care and Use Committee of the Chongqing Medical University (License number: SYXK (Chongqing, China) 2018–0003).

### 2.2. Animal Model and Experimental Protocol

We acquired 12-week-old male C57BL/6 mice, weighing between 22 and 24 g, from the Laboratory Animal Center of Chongqing Medical University (Chongqing, China). All the animals were raised under the following conditions: 25°C, 50 ± 5% humidity, and 12-h/12-h light-dark cycle conditions. The animals were allowed to drink water and eat food freely. Before initiating the study, the mice were raised adaptively for one week.

We used the cecal ligation and perforation (CLP) method in our study, which is the most frequently used method for inducing sepsis. The CLP procedure includes the ileocecal valve ligation post-midline laparotomy and cecal needle puncture. Cecal perforation causes blood polymicrobial infection, which systemically activates the inflammatory reaction that causes a septic shock, ultimately leading to mortality [23]. Briefly, the mice were anesthetized using 100 µL of 20 mg/mL xylazine in PBS and 1 mg/mL ketamine, which was injected intraperitoneally into each mouse. Later, the cecum was ligated and punctured using a 26G needle (nonsevere CLP, inducing 5%–10% mortality among the WT animals). Subsequently, the cecum was returned to the peritoneal cavity, and the incision was closed using surgical staples. Then, to replace the third space loss, the preheated 0.9% saline (37°C) at a concentration of 5 mL/100 g of body weight (BW) was subcutaneously injected into each mouse. After which, a warm pad was prepared for resuscitation.

The article "Exploring the Muscle Metabolomics in the Mouse Model of Sepsis-Induced Acquired Weakness" was published in 2022. Journal: Evid Based Complement Alternat Med.

Both lower limbs were immobilized after surgery. First, one cotton pad was placed near the lower extremities to prevent skin ulceration or compression. Second, the orthopedic casting tape, prepared using a polyester substrate containing the water-activated polyurethane resin (Jinning kangLiDa medical Technology, Shandong, China), was wrapped near the bilateral lower extremities. To minimize the cast movement, mild pressure was applied during the process. Also, chewed plaster, edema, abrasions, and venous occlusions were examined every day once in each animal. However, the activation of the voluntary muscle was not examined. Later, we classified 18 animals into three groups, with six mice in each of the groups. The groups were as follows: normal control, sepsis, and sepsis + AW (acquired weakness, bilateral lower limb-immobilization) groups.

On day 5, ketamine/xylazine mixture was injected into each mouse, and the muscles from the lower bilateral extremity were removed. Later, all muscles were snap-frozen in liquid nitrogen for further testing.

### 2.3. Grip Strength Test

The electronic grip strength meter (Cat.47200, Ugo Basil) was employed to measure the grip strength of the mice. To determine the greatest grip strength, both the lower extremities of the mouse were placed on the fence, which slowly grasped the mouse at its head base.

### 2.4. Assessment of Survival in Mouse Models

To analyze the animal survival, we monitored the survival rate of normal control, sepsis, or sepsis + AW groups of mice for 5 days, with each group having 12 mice.

### 2.5. Transmission Electron Microscopy

After overnight fixation of the muscle samples with 5% glutaraldehyde fixative at 4°C, we cut out the muscle tissues within the identical regions of the two groups into 5-6 tissue blocks (1 mm^3^). Next, the tissue blocks were prepared and observed using transmission electron microscopy (TEM), which was performed at the School of Life Sciences at Chongqing Medical University. Ultrathin sections were prepared as per the previous description [24]. Subsequently, the sections were observed under the TEM (Hitachi-7500, Japan) by a second technician blinded to our experimental protocols. Later, ten fields of view (FOVs) were randomly selected in every section for observation under TEM (magnification, 30,000x).

The article "Exploring the Muscle Metabolomics in the Mouse Model of Sepsis-Induced Acquired Weakness" was published in 2022. Journal: Evid Based Complement Alternat Med.

### 2.6. Muscle Histology

Tibialis anterior muscles were dissected from mice and then immediately dipped into liquid nitrogen for 5–10 seconds and stored at −80°C. In a −20°C cryostat-microtome, tissues were cut in a cross sectional orientation through the muscle mid-belly using a scalpel then embedded in an optimum cutting temperature compound and mounted onto the microtome. Cross sectional cryosections of 10 µm thickness were then taken from the mid-belly of muscle samples, mounted onto glass slides and stored at −20°C.

ATPase activity staining: slides were preincubated at room temperature at pH 4.3 for 5 min, rinsed, and incubated in ATP solution for 25 min. Slides were stained by three washes of 1% calcium chloride solution for 10 min each, incubated in 2% cobalt chloride for 10 min, five exchanges of 5 mM sodium barbital solution, five washes with water, incubated in 2% v/v ammonium sulfide for 20–30 s, and followed by rinsing with five exchanges of water. The slides were dehydrated by ethanol solution incubations and two changes of xylene. The slides were imaged on an microscope system using 20x objective.

COX activity staining: frozen sections were air-dried for 10 to 15 minutes and incubated for 60 minutes in COX staining solution (20 mg/mL catalase, 75 mg/mL sucrose, 2 mg/mL cytochrome C, and 1 mg/mL 3, 3′-diaminobenzidine in 50 mM Na_2_HPO4, final pH 7.4) at 37°C, and then washed in PBS for 2 minutes. The sections were then incubated in SDH staining solution (2 mg/mL Nitrozolium blue tetrachloride), 0.2 M sodium succinate, 50 mM MgCl_2_, 50 mM Tris-HCl, final pH 7.4) for 1 hour at 37°C, and then washed in MQ water for 2 minutes and mounted with glycerol gelatin. The slides were imaged on an microscope system using 20x objective.

### 2.7. Measurement of Inflammatory Mediators

Blood was collected from mice under anaesthesia via the ophthalmic vein into EDTA tubes and then centrifuged at 1,500 rpm for 15 min at 4°C. Serum samples were then divided evenly into the Eppendorf (EP) tubes and preserved at −80°C for subsequent experiments. TNF-*α* (Elabscience, China, #E-EL-M3063), IL-1*β* (Elabscience, China, #E-EL-M0037c), and IL-6 (Elabscience, China, #E-EL-M0044c) in serum were assayed with ELISA kits.

The article "Exploring the Muscle Metabolomics in the Mouse Model of Sepsis-Induced Acquired Weakness" was published in 2022. Journal: Evid Based Complement Alternat Med.

### 2.8. Untargeted Metabolite Extraction

First, we weighed 100 mg (±2%) of samples and added them into the 2 mL EP tube. Next, we added three steel beads and tissue extraction solution (−20°C) (1 mL containing 75% methanol/chloroform mixture (9 : 1, v/v) and 25% H_2_O) into the tubes. Second, the sample was added to the high-throughput tissue grinder and ground at 50 Hz for 60 s, and the process was repeated twice. Later, the samples were subjected to 30-min ultrasonic treatment on ice. Next, the samples were centrifuged at 12000 rpm for 10 min at 4°C. The supernatants (850 µL) were transferred to another 2 mL centrifuge tube and then concentrated and vacuum-dried. The obtained samples were dissolved in 200 µL of 50% acetonitrile solution (containing 2-chlorobenzalanine, 4 ppm), and the supernatants were filtered using the 0.22-µm membrane. Thus, the samples to conduct LC-MS were obtained. Subsequently, 20 µL of the sample was collected to create QC samples, and the deviations in the analytical results from the combined mixed samples were observed. Also, the deviations having errors resulting from the analytical instrument were compared. Further, the remaining samples were collected to conduct LC-MS analysis.

### 2.9. Targeted Metabolite Extraction

#### 2.9.1. Targeted Amino Acid Metabolite Quantification

Ultrahigh-performance liquid chromatography-mass spectrometry (UPLC-MS) analysis of amino acids in mouse muscle was performed on a Waters Acquity UPLC using an ethylene-bridged hybrid (BEH) C18 column (1.7 *μ*m, 2.1 × 100 mm) coupled with a Triple TOF 4000 system equipped with an electrospray ionization (ESI) source operating in negative mode (AB Sciex, USA). Data were analyzed with one-way ANOVA followed by a Tukey post hoc test. First, 23 amino acid standards such as glycine, L-alanine, 4-aminobutyric acid, L-serine, etc., were selected to make standard curve concentrations. Then, 50 milligrams of muscle tissue from mice was weighed, mixed with 600ul of 10% methanol formic acid and 2 glass beads, and shaken for 90s at 60 Hz/s, and this process was repeated at least two times. Next, samples were pulverized by an ultrasonic wave for 30 min and then centrifuged at 12,000 rpm for 5 min at 4°C. 10% methanol formic acid (450 *μ*l) was added after collecting the supernatant (50 *μ*l) and vortexed for 30 s. Finally, we take 100 *μ*L of the sample and add 100 *μ*L of diisotopic internal standard with a concentration of 100 ppb, vortex for 30 s, filter with 0.22 *μ*m membrane, and collect the filtrate for LC-MS analysis.

The article "Exploring the Muscle Metabolomics in the Mouse Model of Sepsis-Induced Acquired Weakness" was published in 2022. Journal: Evid Based Complement Alternat Med.

#### 2.9.2. Targeted Energy Metabolite Quantification

Ultrahigh-performance liquid chromatography-mass spectrometry (UPLC-MS) analysis of energy metabolite in mouse muscle was performed on a Waters Acquity UPLC using an ethylene-bridged hybrid (BEH) C18 column (1.7 *μ*m, 2.1 × 100 mm) coupled with a Triple TOF 4000 system equipped with an electrospray ionization (ESI) source operating in negative mode (AB Sciex, USA). Data were analyzed with one-way ANOVA followed by a Tukey post hoc test. First, 21 energy metabolism standards such as creatinine, PEP, adenosine, cAMP, etc., were selected to make standard curve concentrations. Then, 50 milligrams of muscle tissue from mice was weighed, mixed with 800ul precooled of 80% methanol (−20°C) and 100 mg glass beads, and shaken for 1 min at 55 Hz/s, and this process was repeated at least two times. Next, place the samples in a −20°C ice bath for 40 min. After 40 min, we add 1200 *μ*L precooled of chloroform (−20°C) to the sample, vortex for 30 s, and incubate at 4°C for 10 min. Finally, 1 mL of 0.4 mM ammonia was added, vortexed for 30 s, and incubated at 4°C for 10 min. Then, the content was centrifuged at 12,000 rpm for 10 min at 4°C, then we take 1,500 *μ*L of the supernatant into a 2 mL centrifuge tube, and freeze at −80°C for 3 hours. We reconstitute the sample in 200 *μ*L of the starting mobile phase and collect it for LC-MS analysis.

### 2.10. Liquid Chromatography-Mass Spectrometry Conditions

The ACQUITY UPLC® HSS T3 column (1.8 µm, 150 × 2.1 mm, Waters) was utilized to implement chromatographic separation at 40°C while the temperature of the autosampler was maintained at 8°C. The gradient analyte elution was performed using 5 mM ammonium formate within water (A) and acetonitrile (B) or 0.1% formic acid within water (C) and acetonitrile (D) at a flow rate of 0.25 mL/min for negative and positive ionization, respectively. Every sample (2* µ*L) was injected only upon achieving equilibration. The gradient elution process was as follows: 2% B/D in 0∼1 min, 2%∼50% B/D in 1∼9 min, 50%∼98% B/D in 9∼12 min, 98% B/D in 12∼13.5 min, 98%∼2% B/D in 13.5∼14 min, 2% D-positive model in 14∼20 min (including 2% B-negative model in 14∼17 min).

The ESI-MSn (Thermo, QE–HF–X, USA) assays were conducted at spray voltages of –2.5 kV and 3.5 kV in the negative and positive modes, respectively. Meanwhile, the auxiliary and sheath gases were set at 10 and 30 arbitrary units, respectively, while the capillary temperature was set at 325°C. The range of the full-scan mass analyzer was found to be between 81 and 1000 m/z at a mass resolution of 60000. Later, HCD scans were performed using data-dependent acquisition (DDA) MS/MS analysis. After normalization, the collision energy was set at 30 eV. The redundant MS/MS spectral data were removed using the dynamic exclusion method.

The article "Exploring the Muscle Metabolomics in the Mouse Model of Sepsis-Induced Acquired Weakness" was published in 2022. Journal: Evid Based Complement Alternat Med.

### 2.11. Metabolomic Statistical Analyses

To enable comparison of data of different magnitudes, we batch-normalized the raw data before analysis [25]. The majority of data preserved after the QC, normalization, and QA were used for the analysis. Before analyzing the muscle metabolomics, the Proteowizard software (V3.0.8789) was used to convert the acquired original data to mzXML format (XCMS input file format). Subsequently, *R* (v3.3.2) XCMS package was adopted to determine the identification/alignment/filtration peaks by adopting the following parameters (peak identification: First, we distinguish the entire raw data in the mz dimension to obtain an XIC chromatogram; then, on the basis of each XIC chromatogram, a peak search is performed for the retention time dimension (RT); after that, through the XCMS Algorithms, extract the peak area of the muscle metabolites.): peak width = *c* (10, 20), PPM = 15, bw = 5, mzdiff = 0.01, mzwid = 0.015, and method = centWave. Next, the data matrix, including the intensity, retention time (RT), and mass-to-charge ratio (M/Z), was acquired, and the data were exported into an Excel sheet (using HMDB, massbank, lipidmaps, mzcloud, KEGG databases to identify substances). Furthermore, the obtained data were subjected to autoscaling and mean-centering and were scaled to unit variance (UV) before multivariate statistical analysis to obtain more reliable and intuitive results. Subsequently, the resultant data were fed to *R* package Ropls (R language ropes package [26]) for multivariate principal component analysis (PCA), partial least-square discriminant analysis (PLS-DA), and orthogonal partial least-square discriminant analysis (OPLS-DA). Additionally, to compare the data of diverse orders, normalized peak area data were batched.

### 2.12. Other Statistical Analyses

SPSS 22.0 was adopted to perform statistical analysis. All the data were represented as mean ± SD unless indicated otherwise. To compare between the several groups, the Kruskal–Wallis one-way analysis of variance followed by the Mann–Whitney *U* test for post hoc comparisons were performed. Survival curves were assessed by the log-rank (Mantel–Cox) test. Differences between and among groups were considered to be statistically significant at *P* < 0.05.

## 3. Results

### 3.1. The Effects of Muscle Injury during Sepsis-AW

The experimental model of sepsis-acquired muscle weakness in C57BL/J mice was constructed according to the research method of Bassem Habr et al. To evaluate the effect of the model, we first measured the weight of the bilateral lower limb muscles of mice from each experimental group. The results showed that compared to the healthy control and sepsis group, a significant reduction was observed in the muscle weight of the lower limb of the mice with sepsis-acquired muscle weakness (sepsis-AW group) after 5 days modeling (Figure 1(a)). With the extension in the model time, the grip strength of the lower limb muscles showed a gradual decrease. By the 5th day of modeling, the grip strength of the mice reached the lowest (Figure 1(b)). In addition, there is no significant difference in the survival rate of mice in each experimental group (Figure 1(c)). In order to verify the systemic inflammation intensity in each experimental group, we measured the inflammatory mediators, such as TNF-*α*, IL-1*β*, and IL-6, in the mouse serum by an ELISA kit. On the fifth day of modeling, the levels of IL-1*β*, IL-6, and TNF-*α* in the mouse serum were not significantly different between the sepsis and sepsis-AW group but were significantly higher than those in the normal control group (Figure 1(d)). After 5 days of modeling, the transmission electron microscopic images showed more clear evidence of swollen mitochondria and disordered arrangement of myofilaments in the muscle tissues of the sepsis-AW group (Figure 1(e)). Besides, the sepsis and sepsis-AW models mainly affect type I muscle fibers in the lower limbs of mice as indicated by ATPase staining (Figure 1(f)). More importantly, it affects the mitochondrial function in type I muscle fibers (Figure 1(g)).

The article "Exploring the Muscle Metabolomics in the Mouse Model of Sepsis-Induced Acquired Weakness" was published in 2022. Journal: Evid Based Complement Alternat Med.

### 3.2. The Chromatogram in the Total Ion Mode

The chromatography-separated components were analyzed using mass spectrometry (MS), and the data were collected continuously through the scanning mass spectra. The time and intensity were plotted as abscissa and ordinate, respectively. The formed spectrum represented the base peak chromatogram (BPC), which is shown in Figures 2(a) and 2(b) (1: normal control group, 2: sepsis group, and 3: sepsis-AW group).

### 3.3. Analysis of Muscle Metabolomics in Positive- and Negative-Ion Mode

During the preprocessing of data (format transformation, peak recognition, and normalization, along with filtering alignment), we selected the highly repeatable data facilitating positive-/negative-ion mode muscle metabolomics analysis. Following the data preprocessing, the principal component analysis (PCA) was performed to explore the muscles in sepsis-AW mice in both modes. The alterations in metabolic profiles generated a model containing two principal components (*R*2 = 0.522cum and *R*2 = 0.546cum for negative and positive, respectively) and one score chart reflecting intergroup dispersion level (Figure 2(c)). As exhibited by the PCA score diagram, a majority of samples lay within the 95% CI ellipse, except for several outliers. Based on the PCA score diagram, the muscle samples from all three groups showed marked differences with statistical significance. Additionally, the OPLS-DA and PLS-DA approaches (Figures 2(d) and 2(e)) were used to remove the data irrelevant to sample classification. Next, pattern discrimination was applied in the full spectrum of muscles. Altogether, 200 PLD-DA permutation tests were conducted, and it was found that R2 and Q2 in the positive-ion mode were (0.0, 0.95) and (0.0, -0.03), respectively, while those in the negative-ion mode were (0.0, 0.96) and (0.0, 0.13), respectively. As a result, all three groups showed marked differences. To check whether our model was repeatable and to ensure that our data were reliable, we further conducted a permutation test on the model (Figure 2(f)), and as a result, we found that the muscle sample multivariate data model satisfied the parameter standards indicating its high stability and predictability.

The article "Exploring the Muscle Metabolomics in the Mouse Model of Sepsis-Induced Acquired Weakness" was published in 2022. Journal: Evid Based Complement Alternat Med.

### 3.4. Extraction and Analysis of Differential Metabolites

Consistent screening thresholds were applied in the PCA, OPLS-DA, and PLS-DA in all the three groups, with VIP ≥ 1 and *P* value ≤ 0.05. In the positive-ion mode, 2630 upregulated and 3812 downregulated features were found in the sepsis group compared to the normal group. Similarly, in the sepsis-AW group, 2741 upregulated and 3408 downregulated features were observed. Compared to the sepsis group, the sepsis-AW group showed 823 upregulated and 566 downregulated features (Figure 3(a)). Compared to the normal group, the sepsis group showed 1548 upregulated and 2190 downregulated features in the negative-ion mode, while the sepsis-AW group showed 2851 upregulated and 1038 downregulated features. Compared to the sepsis group, the sepsis-AW group showed 1952 upregulated and 391 downregulated features (Figure 3(b)). Based on the fragmentation data acquired in the MS/MS mode, more matching annotations were obtained from METLIN, mzCloud, HMDB, LipidMaps, and MassBank databases to determine the precise identity of metabolites. Altogether, 84 differentially genes are expressed metabolites (DEMs), including 35 upregulated and 49 down-regulated metabolites, with similar or consistent metabolic modes that were classified to obtain the heatmap for differential metabolites (Figure 3(c)). The above differentially expressed metabolites were identified from different databases, including KEGG, Marker-view, MetaboAnalyst, and HMDB (Table 1). Further in-depth analysis showed that among the 84 different metabolites, 30 metabolites were observed in the sepsis and sepsis-AW groups, of which 17 were upregulated and 13 were downregulated (Figure 3(d)).

The article "Exploring the Muscle Metabolomics in the Mouse Model of Sepsis-Induced Acquired Weakness" was published in 2022. Journal: Evid Based Complement Alternat Med.

### 3.5. Information on the Differential Metabolic Pathways in the Muscles of the Sepsis-AW Mouse Model

In the present study, DEMs were aligned against the KEGG database. The DEMs from the sepsis group and the sepsis-AW group were found to be enriched in 54 metabolism-related pathways, which is shown in Figure 4. Of these pathways, valine/leucine/isoleucine biosynthesis, purine metabolism, cGMP-PKG pathway, mTOR pathway, FoxO pathway, and PI3K-Akt pathway satisfied the conditions of Impact > 0.2 and *P* < 0.05. The main metabolites involved in these metabolic pathways included Leu, AMP, 2-oxobubanoate, cAMP, GMP, and adenylosuccinate, which are listed in Table 2.

### 3.6. Analysis of Target Amino Acids and Energy Metabolites

In the second step of our metabolomic investigation, we used targeted metabolomics to quantify 22 amino acid metabolites and 20 energy metabolites in the muscle samples. In the quantitative analysis of targeted amino acid metabolites, compared to the sepsis group, the sepsis-AW group showed a significant increase in four metabolites (leucine, cysteine, tyrosine, and serine). However, the other 18 amino acid metabolites did not show any significant changes between the two groups (Figures 5(a)-5(b)). In the quantitative analysis of 20 energy metabolites, the level of one energy metabolite (AMP) was found to be elevated, while the level of another energy metabolite (cAMP) was found to be lowered (Figures 5(c)-5(d)).

## 4. Discussion

Intensive care unit-acquired weakness (ICU-AW) refers to “the weakness of critical patients with no other plausible etiology, except, the critical disease during the clinical treatment” [27]. As early as the 19th century, scholars discovered that the loss of muscles caused by ICU-AW could directly threaten a patient's life. ICU-AW in critical patients has been associated with sepsis, acute respiratory distress syndrome, and multiple organ dysfunction syndrome as prevalent complications [13]. Sepsis can cause crucial organ dysfunction of the heart, kidney, or liver, which might directly threaten the patients' survival [28]. However, the mid-long-term recovery of the patients was obstructed by the continuous failure of vital organs, usually along with the nonvital organs, such as the skeletal muscle [29]. Sepsis accompanying skeletal muscle dysfunction (locomotive or respiratory) can intensify a feed-forward paresis-infection cycle, ultimately causing death [3]. During sepsis, the inflammatory response gets out of control, which is accompanied by the release of a large number of inflammatory factors [30]. The levels of the release of cellular inflammatory factors (TNF-*α*, IL-6, IL-1, and IFN-*γ*) are closely related to the muscle mass (loss of imbalance between protein synthesis rate and degradation) [31]. The most popular reason behind the origin of sepsis-induced myopathy is attributed to circulating pathogens and cytokines related to halted protein synthesis (due to overproduction of reactive oxygen species) and accelerated protein degradation (due to reinforced proteasome proteolytic degradation and autophagy pathways) [32]. The results hinted that the continuous and unopposed inflammatory processes in sepsis encouraged TNF-*α* production along with corresponding catabolic effects against the murine skeletal muscle [33]. This decreased mitochondrial respiration and impaired biogenesis (via PGC-1*α* inactivation) [34]. Besides, the sepsis-induced ischemia/hypoxia injury, protease system activation and oxidative stress can lead to changes in the ion channels, which is the basis of neuromuscular diseases [35]. Moreover, sepsis also caused mitochondrial dysfunction central to muscle disuse atrophy [36]. Thus, sepsis-induced muscle weakness involved changes in energy homeostasis as well as muscle protein catabolism. Previous studies have shown that metabolomics can identify metabolites in biological systems [37]. The characteristics of metabolites can help in predicting the high-risk factors for the disease along with providing stratification of disease severity. This leads to an improved understanding of disease mechanisms [38]. In our research, multiple methods such as statistics, bioinformatics, and chemometrics, including the PCA, PLS-DA, and OPLS-DA diversified analysis, were employed to analyze and compare the differential metabolites. Significant metabolic differences were found in the mice muscles between the sepsis and sepsis-AW groups. Metabolomic untargeted assay (from Kyoto Encyclopedia of Genes and Genomes (KEGG) data) (*P* < 0.05 and impact > 0.2) was used to identify 30 different metabolites and six metabolic pathways. The results showed the presence of multiple types of differential metabolites in sepsis-AW group, potentially corresponding to different predictable metabolic pathways. However, recognizing the commonalities among numerous metabolites and metabolic pathways remains a contemplative process.

The article "Exploring the Muscle Metabolomics in the Mouse Model of Sepsis-Induced Acquired Weakness" was published in 2022. Journal: Evid Based Complement Alternat Med.

First, the amino acid metabolic processes involving multiple molecules and biochemical metabolic pathways may show changes during the occurrence of sepsis-AW. According to the high-throughput MS, four amino acids (leucine, cysteine, tyrosine, and serine) were found to be significantly increased during the sepsis-AW. Previous studies have proven that leucine plays a key role in regulating global protein synthesis while maintaining cellular protein homeostasis through the promotion of mammalian target of rapamycin (mTOR) activity [39]. Also, the cysteine-rich domains are found to control protein synthesis, reduce muscle mass loss, and regulate skeletal muscle function [40]. Cysteine's role in treating sepsis and promoting survival rates has been verified by clinical and animal investigations [41]. The release levels of tyrosine in muscle proteins can be used as the indicator to estimate the degree of endotoxin-induced proteolysis and muscle mass of the diaphragm along with lesser levels of protein content in the total diaphragm [42]. Experimental animal studies have also confirmed that serine may effectively reduce the accumulation of increased ROS in the mouse skeletal muscle. This increases the antioxidant enzyme activity and protects the mice from oxidative stress-induced muscle weakness [43]. These findings suggested that protein metabolism is a depleting process in sepsis-AW. In the case of sepsis-induced acquired weakness, leucine, cysteine, tyrosine, and serine may be considered more sensitive biomarkers.

Second, the essence of sepsis is considered to be the abnormal metabolism of cellular energy [28]. During sepsis, mitochondria, the main site of systemic oxygen consumption, may play a role in consuming excessive oxygen and creating “cytopathic hypoxia” [44]. When sepsis occurs, the body reduces the mitochondrial respiratory chain function, which is accompanied by free radical generation and bioenergetics reprogramming of glycolytic metabolism [20]. Innovative research by Mervyn Singer's laboratory claimed that after 24 h of ICU admission of the septic shock patients, their skeletal muscle biopsies showed severely damaged mitochondrial ETC [45]. Similarly, in a recent human quadriceps comparative research on mitochondrial respiration dysfunction, Jiroutková et al. observed that compared to the controls, the muscles of septic patients showed functional impairments and quantitative defects in their respiratory complexes [44]. Thus, energy metabolism played an important role in sepsis-acquired weakness. To regulate energy homeostasis and signal transduction, adenosine monophosphate (AMP) played an important role in the production of cellular metabolites [46, 47]. Earlier studies have found that systemic hypoxia can cause an increase in AMP, ADP, and other energy metabolites in the homogenate samples of the skeletal muscles [48]. Intercellular AMP is critical for reprogramming metabolism and regulating growth, which happens through the activation of AMP-activated protein kinases (AMPKs) [49]. AMPK, an important sensor for cellular energy status, can regulate cellular metabolism and maintain energy homeostasis [50]. Studies have shown that in myopathy or in myopathy that includes muscle weakness, atrophy, and other diseases, downregulation of AMP-activated protein kinase (AMPK) may lead to an increase in autophagy, apoptosis, and ubiquitin-proteasome activity, ultimately causing muscular dystrophy [51]. However, AMPK consists of sites that reversibly bind to AMP or ATP, switching on the kinase along with increasing the cellular AMP : ATP ratio (indicating lowered cellular energy status). Upon activation, AMPK can switch on the catabolic processes producing ATP, which simultaneously switches off unnecessary energy-requiring processes in the short run [52]. Hence, it can acutely activate glucose uptake and fatty acid oxidation while simultaneously switching off glycogen and protein synthesis (through inactivation of the mammalian target-of-rapamycin pathway) [53, 54]. Therefore, AMPK activation is also considered an adaptive mechanism in response to sepsis [55]. Cyclic adenosine monophosphate (cAMP) is the main molecule that regulates cell metabolism and biological functions and is also called the “second messenger” during the transmission of life information [56]. Many physiological processes of the vertebrate skeletal muscle can be regulated via the cAMP-dependent intracellular signaling pathways such as muscle differentiation, metabolism, or contraction. In the skeletal muscle, cAMP signaling was related to the regulation of glycogenolysis [57], contractility [58], sarcoplasmic calcium dynamics [59], and also to the recovery from continuous contractile activity [60]. Nevertheless, numerous surveys have indicated that cAMP-inducing agents or genetic modifications of the proteins of cAMP signaling may generate adaptive effects on the skeletal muscle through amplification of myofiber size, facilitating fiber-type transfer to glycolytic fibers [61–63]. Grossman et al. found that insufficient cAMP levels may lead to cardiac and skeletal muscle dysfunction [64]. The cAMP signaling is involved in the differentiation [65], migration [66], and fusion of muscle precursor cells [67]. In an adult muscle, the stimulation of cAMP production slows the degeneration or promotes the regeneration of rodent muscles during necrotic muscle injury [66] and Duchenne's muscular dystrophy [57, 68]. We studied and found an obvious increase in AMP and a decrease in cAMP levels in the septic myasthenia mouse model. However, other energy metabolites did not show significant changes. These findings suggested that both AMP and cAMP metabolism levels may serve as potential biomarkers in the diagnosis of sepsis-acquired weakness.

The article "Exploring the Muscle Metabolomics in the Mouse Model of Sepsis-Induced Acquired Weakness" was published in 2022. Journal: Evid Based Complement Alternat Med.

Third, the current research also explored metabolic pathways mainly through the KEGG data. According to our research, an increase was observed in both amino acid metabolism and energy expenditure in the mouse model of sepsis-AW (based on our results). Significant differences were observed in the metabolic signaling pathways, including the mTOR, PI3K/AKT, and FoxO pathways, between the sepsis and sepsis-AW groups. The skeletal muscle mass is regulated by a complex set of signaling pathways [69]. In most cell types, the kinase mTOR is the main regulator of cellular metabolism, protein synthesis, or turnover [70]. In the skeletal muscle, pharmacological and genetic interventions affect the mTORC1 signaling pathway and indicate the significant impacts of modulation of the complex's activity on the increased size and function of the muscle [71]. Besides the regulation of increased protein synthesis, many studies also associated mTORC signaling with protein breakdown [72]. Previous research studies have demonstrated that enhanced autophagic flux in the adult skeletal muscle during catabolic conditions is primarily regulated through FoxO transcription factors [73], while basal autophagy is regulated through mTORC signaling [74]. Upon the removal of the kinase mTOR from the skeletal muscle, a similar late-onset of myopathy was observed, which was accompanied by premature death [75]. Hence, the maintenance of the neuromuscular junction requires mTORC1 signaling in the muscle tissues. Long-term inhibition of mTORC1 signaling can cause myopathy [70]. A study showed that testosterone propionate promoted the phosphorylation of the mTOR signaling pathway, improving the strength, endurance, and volume of the skeletal muscle in septic rats [76]. Protein degradation in the skeletal muscle is similar to that of the mammalian cells and is under the control of two main proteolytic systems, including ubiquitin-proteasome and autophagy-lysosome [77]. The degradation pathways can be activated by diverse catabolic diseases, such as cancer, AIDS, diabetes, or heart and renal failure. This can lead to loss and weakness of the muscles [78]. In the skeletal muscle, both these systems are regulated by the FoxO pathway. However, their excessive activation may induce serious muscle loss [79]. FoxOs modulate the catabolic processes involving VIDD—UPS, autophagy, and apoptosis. Specifically, FoxOs directly activate atrophic genes such as MAFbx/Atrogin-1 and MuRF1 along with an autophagy marker gene LC3 [80]. FoxOs facilitate apoptotic signaling via the induction of several members of the Bcl2 family (such as apoptosis facilitator gene Bim/Bcl2 l11 that modulates the permeability of mitochondrial membrane) along with stimulation of the expression of death receptor ligands, including the Fas ligand. Furthermore, the FoxOs modulate the mitochondrial function and glucose metabolism, possibly by serving as the “dysfunction” component during the VIDD. For instance, FoxO3a can regulate glycolysis and decrease DNA copy number, proteins, and respiratory activity in the mitochondria [81]. A FoxO blockade that uses a dominant-negative FoxO is known to prevent VIDD. Consequently, screening metabolic pathways can help in assessing metabolic changes during sepsis.

The article "Exploring the Muscle Metabolomics in the Mouse Model of Sepsis-Induced Acquired Weakness" was published in 2022. Journal: Evid Based Complement Alternat Med.

## 5. Conclusion

Metabolomics presents a major technique in the study of disease pathogenesis and diagnosis. First, our study used LC-MS metabolomics to diagnose sepsis-AW, which was based on muscle metabolites. Combining PCA with supervised analysis methods such as PLS-DA and OPLS-DA can help in recognizing differential metabolites in the model and the control groups. Our study found such differences primarily among 30 metabolites and six different metabolic pathways. Targeted analysis of metabolomics can be used to identify amino acid metabolites, including leucine, cysteine, tyrosine, and serine as well as energy metabolites, including AMP and cAMP, which in turn, can be used as biomarkers for the diagnosis of sepsis-AW.

## Figures and Tables

**Figure 1:** The C57BL/5 mice were classified into the following three groups: the no-treatment group (normal control group), the sepsis model group, and the sepsis-AW model group, with six mice in each group. The representative plots are shown as follows. (a) Mass variation diagram of the lower limb muscles and body weight of the normal control group, sepsis group, and sepsis-AW group. (b) The grip strength of the lower limb muscles computed using an electronic grip strength meter. (c) Mouse survival (*n* = 12 mice/group) were assessed by the log-rank test. (d) Cytokines level (IL-1*β*, IL-6, TNF-*α*) in the serum in mice were measured by the mouse cytokine ELISA kit at 5 d following modeling. (e) The morphological changes in the lower limb muscles of the mice in each group observed using transmission electron microscopy. (f, g) ATPase and COX staining of tibialis anterior muscles groups from normal control, sepsis, and sepsis-AW group.

**Figure 2:** (a, b) Each line represents a typical sample-based peak chromatogram in both positive- and negative-ion mode (1: normal control group, 2: sepsis group, and 3: sepsis-AW group). (c–f) Metabolism profile of the muscles in the sepsis-AW mouse model in positive- or negative-ion mode including PCA, PLS-DA, OPLS-DA scores, and the replacement test of the muscles fit model in positive- or negative-ion mode in the sepsis-AW group.

The article "Exploring the Muscle Metabolomics in the Mouse Model of Sepsis-Induced Acquired Weakness" was published in 2022. Journal: Evid Based Complement Alternat Med.

**Figure 3:** (a, b) Statistical findings of differential metabolites in positive- or negative-ion mode. (c) Heat map of differential metabolites in the normal control, sepsis, and sepsis-AW groups. (d) Heat map of the differential metabolites in the sepsis and sepsis-AW group.

**Figure 4:** Metabolic pathways in the sepsis-AW mouse model mapped to KEGG.

**Figure 5:** C57BL/5 mice were divided into the following three groups: no-treatment (normal control group), sepsis, and sepsis-AW groups, with six mice in each group. (a) The heat map of 22 amino acid differential metabolites in the muscle samples of the normal, sepsis, and sepsis-AW groups as measured using targeted metabolomics. (b) Increased levels of leucine, cysteine, tyrosine, and serine as observed in the muscle of the sepsis-AW group mice. (c) The heat map of 20 energy differential metabolites in the normal, sepsis, and sepsis-AW muscle samples measured using targeted metabolomics. (d) Enhanced levels of AMP and reduced levels of cAMP observed in the muscles of the sepsis-AW group. ^*∗*^*P* < 0.05, ^*∗∗*^*P* < 0.01, and ^*∗∗∗*^*P* < 0.001 through the Kruskal–Wallis one-way analysis of variance followed by the Mann–Whitney *U* test for post hoc comparisons represent comparison between the control, sepsis, and sepsis-AW groups.

**Table 1:** Differential metabolic markers in the muscle of sepsis-AW mouse.

IDs	Chemical compound	VIP	*P* value
C01367	3-AMP	1.98568	2.16E-05
C07073	Lidocaine	2.12969	2.26E-05
C02115	2-Methylserine	1.00063	7.53E-05
C02043	Indolelactic acid	2.00667	0.00016
C21308	(S)-Beta-tyrosine	2.12782	0.00018
C00345	6-Phosphogluconic acid	1.66238	0.00028
C03440	cis-4-Hydroxy-D-proline	1.76335	0.00034
C00123	L-Leucine	2.02159	0.00044
C04741	Prostaglandin E1	1.72049	0.00069
C00021	S-Adenosylhomocysteine	1.74668	0.00077
C02752	Triacetate lactone	1.89111	0.00095
C03030	Uracil 5-carboxylate	1.94223	0.00096
C11016	Diphenylamine	1.17166	0.00101
C02183	Phloroglucinol	1.21557	0.00170
C11963	Avermectin B1b aglycone	1.71957	0.00175
C02846	N, N-Dimethylaniline	1.92473	0.00230
C12270	N-Acetylaspartylglutamic acid	1.41928	0.00324
C03431	S-Inosyl-L-homocysteine	1.83690	0.00516
C00188	L-Threonine	1.61459	0.00524
C05572	4-Oxoglutaramate	1.80158	0.00619
C07474	Pilocarpine	1.81274	0.00625
C00811	4-Hydroxycinnamic acid	1.48410	0.00647
C07577	3, 4-Methylenedioxyamphetamine	1.25536	0.00663
C05318	cis-N-Methyl-(S)-7, 8, 13, 14-tetrahydroprotoberberine	1.51731	0.00711
C03451	S-Lactoylglutathione	1.76992	0.00725
C07276	Limonene-1, 2-diol	1.75758	0.00807
C06413	Quinoline	1.32957	0.00923
C01746	Piperidine	1.31122	0.01150
C02700	L-Formylkynurenine	1.34456	0.01193
C07868	Metoclopramide	1.36527	0.01211
C03794	Adenylsuccinic acid	1.50630	0.01217
C20579	Cyclopeptine	1.68896	0.01292
C00534	Pyridoxamine	1.71393	0.01308
C00147	Adenine	1.53898	0.01452
C10761	p-Anisaldehyde	1.67325	0.01480
C01733	Racemethionine	1.23461	0.01565
C00931	Porphobilinogen	1.54395	0.01571
C00255	Riboflavin	1.60986	0.01574
C06951	Dicyclomine	1.58051	0.01698
C00294	Inosine	1.60000	0.01888
C05584	Vanillylmandelic acid	1.46427	0.01986
C02632	Isobutyric acid	1.47142	0.02062
C00449	Saccharopine	1.57923	0.02101
C00380	Cytosine	1.54665	0.02187
C00526	Deoxyuridine	1.63133	0.02246
C00049	L-Aspartic acid	1.43749	0.02852
C01234	1-Aminocyclopropanecarboxylic acid	1.30302	0.03189
C02679	Dodecanoic acid	1.48122	0.03535
C08679	Deltaline	1.47756	0.03587
C00378	Thiamine	1.44937	0.04049
C00073	L-Methionine	1.20471	0.04098
C02587	Pyrimidodiazepine	1.39701	0.04154
C02486	Beta-Leucine	1.46871	0.04424
C00135	L-Histidine	1.48382	0.04505
C01179	4-Hydroxyphenylpyruvic acid	1.07514	0.04508
C05527	3-Sulfinylpyruvic acid	1.46882	0.04634
C11171	Sodium deoxycholate	1.49561	0.04860
C00296	Quinate	2.23964	0.00006
C01586	Hippuric acid	1.98906	0.00160
C18319	Ethylmethylacetic acid	1.91831	0.00268
C02727	N6-Acetyl-L-lysine	1.78134	0.00302
C14775	14, 15-DiHETrE	1.64533	0.00637
C14871	S-(Formylmethyl) glutathione	1.47199	0.00698
C00233	Ketoleucine	1.73028	0.00705
C01073	N-Acetyl-beta-alanine	1.22414	0.00840
C05283	N2-Gamma-glutamylglutamine	1.83316	0.00890
C19615	Hexadecanedioate	1.47617	0.01143
C05598	Phenylacetylglycine	1.22311	0.01449
C05332	Phenylethylamine	1.77227	0.01515
C00120	Biotin	1.55771	0.01618
C00847	4-Pyridoxic acid	1.67106	0.01742
C00025	L-Glutamate	1.59469	0.01954
C06196	dIMP	1.56779	0.02035
C05512	Deoxyinosine	1.58788	0.02492
C07588	Salicyluric acid	1.57050	0.02643
C00310	L-Ribulose	1.33197	0.02651
C08278	Suberic acid	1.62103	0.03200
C01762	Xanthosine	1.62912	0.03235
C16511	L-Homocysteic acid	1.11491	0.03883
C00301	Adenosine diphosphate ribose	1.34036	0.03906
C00149	L-Malic acid	1.52310	0.04263
C00232	Succinic acid semialdehyde	1.49534	0.04293
C00669	Gamma-glutamylcysteine	1.56048	0.04539
C00031	D-Glucose	1.54665	0.04725

The article "Exploring the Muscle Metabolomics in the Mouse Model of Sepsis-Induced Acquired Weakness" was published in 2022. Journal: Evid Based Complement Alternat Med.

**Table 2:** Differential metabolic pathways in the muscle of sepsis-AW mouse.

<!—Col Count:7	Total	Hit	Raw *P*	Log (*P*)	Impact	Compounds
mTOR signaling pathway	4	2	0.000469	7.6632	0.5	Leu and AMP
Valine, leucine, and isoleucine biosynthesis	23	2	0.017804	4.0283	0.33	Leu and 2-oxobubanoate
cGMP-PKG signaling pathway	10	2	0.003406	5.6821	0.28571	AMP and cAMP
Purine metabolism	95	3	0.033991	2.9381	0.23	AMP, GMP, and adenylosuccinate
PI3K-Akt signaling pathway	4	1	0.035727	3.3319	0.2	AMP
FoxO signaling pathway	5	1	0.044464	3.1131	0.2	AMP

## Data Availability

The datasets used or analyzed during the current study are available from the corresponding author on reasonable request.
